# Construction of a Meta-Evidence Prototype Database of Traditional Chinese Medicine Splenogastric Diseases and Its Application in an Automatic Meta-Analysis System

**DOI:** 10.1155/2022/6933523

**Published:** 2022-07-13

**Authors:** Xueqin Zhang, Chunying Wang, Yanning Yao, Wenyu Sun, Yujie Guo, Lin Ma, Xinyuan Lu, Hongyong Deng

**Affiliations:** TCM Science and Technology Information Center, Shanghai University of Traditional Chinese Medicine, Shanghai, China

## Abstract

**Background:**

Traditional Chinese medicine splenogastric diseases (TCMSDs) are equivalent to digestive system diseases in modern medicine. The forms of clinical evidence of TCMSDs include clinical trials, such as randomized controlled trials (RCTs) and systematic reviews (SRs). SRs mainly rely on manual operations and have the shortcomings of time consumption and low efficiency; therefore, they cannot meet the needs of rapid clinical decision-making. It is urgent to establish a new and smart form of a database to support the progress of SRs.

**Methods:**

We searched and screened all TCMSD RCT reports, in both Chinese and English, and extracted them into meta-evidence through predesigned structural Microsoft Excel tables. All meta-evidence was imported into an online clinical meta-evidence collection and management system after data quality checking. The meta-evidence database of traditional Chinese medicine (TCM) splenogastric disease (MED-TCMSD) was then tested as a backend of an automatic meta-analysis system.

**Results:**

A total of 405 cases of TCMSD RCTs were processed into meta-evidence. The most common diseases were stomach stuffiness disease, epigastralgia, and chronic atrophic gastritis. Banxiaxiexin decoction and its modifications were the most used interventions. More than half of the cases employed TCM in conjunction with regular therapeutics. The top reported outcomes included clinical effects, adverse events, and TCM syndromes. The MED-TCMSD worked well as a part of the automatic meta-analysis system.

**Conclusions:**

We developed and tested a new form of clinical evidence, meta-evidence, for automatic SR and fast evidence-based decision-making. As an example of the MED, the MED-TCMSD can improve the production and updating efficiency of the evidence of TCMSDs. The methods of constructing the MED-TCMSD can be further applied to the development of MEDs of other diseases.

## 1. Introduction

Traditional Chinese medicine splenogastric diseases (TCMSDs) are a variety of diseases and symptoms that are related to gastrointestinal functions. Their clinical incidence rate is relatively high. For example, the prevalence of functional dyspepsia in China is 7%–41%, the prevalence of irritable bowel syndrome in China is 5%–25% [1], and the prevalence of gastrointestinal diseases in urban adults is 17.41% [2]. There are numerous therapeutics for these conditions in clinical practice, which can be grouped into three classes: traditional Chinese medicine (TCM) (e.g., TCM decoction [3], Chinese patent medicine [4], and acupuncture [5]), integrated traditional Chinese and Western medicine [ITCWM]) [6, 7], and Western medicine [8]. To help doctors deal with the complicated and variable clinical conditions of TCMSDs quickly and accurately, many scientific research teams have built different kinds of splenogastric disease databases. For example, Huang [9] constructed an online database of irritable bowel syndrome (IBS) with functions of patient data management, statistics, analysis, and data mining. Chen [10] created a database of TCM clinical support for *H. pylori* infection-related diseases. Chen [11] constructed a chronic gastritis database for the diagnosis and treatment of ITCWM. With the help of the databases, retrospective research can be carried out to explore the connections between TCM and Western medicine. Yan et al. [12] established an online database of the transcriptome of IBS, which integrated and stored 320 IBS gene samples in the Gene Expression Omnibus and ArrayExpress databases. By allowing comparisons of the gene expression levels of IBS patients, this database can help the exploration of the pathogenesis of IBS and the development of drugs. Khanna et al. [13] developed the GI-PRO database, which is an online library of patient-reported outcome measures in gastroenterology. This database can guide clinical decision-making, research, and drug approval. However, most of these databases only include patient case information, and although they can provide a reference for clinical activities, they have limited value in supporting evidence-based clinical decision-making [14, 15]. Therefore, there is a need for databases that can directly support clinicians.

Evidence-based medicine (EBM) databases can be classified into four types [16]: clinical practice guideline (CPG) databases, systematic review (SR) databases, clinical trial databases, and comprehensive EBM databases. They differ in their objective, scope, content, and service target groups but share the same foundations as SRs. The typical processes of SRs include protocol writing, study retrieval, data extraction, evidence synthesis, and evidence evaluation, which are mainly performed manually and are frequently lengthy and inefficient undertakings. The abovementioned four kinds of EBM databases are currently fully developed and have been applied in clinical decision-making. However, they are not designed for rapid evidence-based decision-making based on automatic SRs (ASRs). ASRs employ computer automation techniques, such as natural language processing, text mining, and machine classification, in all phases of an SR to optimize its procedures and improve its efficiency [17, 18]. Data are the essential part of an ASR system. The efficiency requirements of ASRs call for a new form of evidence database besides the current four types of EBM databases.

In this study, we explored a kind of clinical evidence database that is highly standardized and structured to meet the needs of automatic systematic reviewing. We named it the meta-evidence database (MED). It is pre-extracted and stored in a machine-readable data format. We constructed a MED of TCM splenogastric disease (MED-TCMSD) and implemented it in a fast evidence-based decision-making system based on ASRs to test its functions and advantages.

## 2. Methods

### 2.1. Data Sources

#### 2.1.1. Databases and Retrieval Strategy

The literature databases that we referred to were four Chinese databases (CNKI, WanFang Data, VIP, and SinoMed) and four English databases (PubMed, Cochrane Library (CENTRAL), Web of Science, and Ebsco Medline). Each database was searched separately for TCM splenogastric disease randomized controlled trials (RCTs) without any time limitations. The search terms were RCT, randomized controlled trial, and a group of specific disease names. We identified 12 TCM diseases corresponding to TCM splenogastric disease: epigastralgia, acid regurgitation, epigastric upset, stomach stuffiness disease, vomiting, hiccup disease, dysphagia disease, regurgitation disease, abdominal pain, diarrhea disease, constipation disease, and dysentery.

#### 2.1.2. Inclusion and Exclusion Criteria

The inclusion and exclusion criteria followed the patient/population, intervention/exposure, comparison/control, outcome, and study design (PICOS) rule [19]. The inclusion criteria were the following: patients diagnosed with TCM splenogastric disease, namely the abovementioned 12 diseases (see 2.1.1); interventions of TCM alone (TCM interventions included herbs, massage, qigong, acupoint-pressing, and acupuncture) or TCM combined with Western medicine; blank control, placebo control, or positive control (add-on study); all outcomes; RCT study design. The exclusion criteria were the following: animal experiment or in vitro experiment; Western medicine-only intervention; non-RCT study design, semi-random, or pseudo-random studies; duplicate literature.

#### 2.1.3. Literature Screening

The screening process was carried out independently by two researchers in three steps: (1) Search results were imported and automatically screened in NoteExpress software to remove the duplicates; they were rechecked manually. (2) The abstracts of the papers were examined carefully according to the selection criteria. Most exclusions were carried out for reasons in this step. (3) The last step was to check all the remaining full texts to make the final inclusion. Two authors completed the screening independently and cross-checked the results for correctness.

### 2.2. Data Extraction

#### 2.2.1. Extraction Table

A standardized extraction table can facilitate the extraction of data. We created a data sheet for extraction based on Microsoft Excel powered with Visual Basic for Applications (VBAs). The extraction tables of the clinical evidence were designed for data collection, which can be imported into the database in the batch mode. The VBA code built in the table can enable basic data inspection and verification of the input data. Each study was assigned a unique number to identify while storing and citing. The full texts (PDF) of the included studies are attached for reference.

#### 2.2.2. Extracting Content and Methods

Based on the characteristics of RCTs, the extraction table contained six sections: general information, evidence sources, clinical data, trial design, grouping and interventions, and outcomes. (1) The general information section has 10 fields, such as evidence ID, evidence status, creation time, evidence name, clinical trial register number, data editor, and reviewer. (2) The evidence sources section has 24 fields, such as source type, article title, journal source, author information, author institution, contact information, grant number, and DOI and full-text path or link. (3) The clinical data section has 23 fields, such as diagnosis (both TCM and Western medicine), sample size, age and gender, course of the disease, inclusion criteria, and exclusion criteria. (4) The trial design section has 19 fields, such as study type, randomization type, blindness type, observation time, and risk of bias factors (randomization, allocation concealment, blinding, missing data, selective reporting, and other bias). (5) The grouping and intervention section has 27 fields, such as group name, sample size of each group, age and gender of each group, observation/control type, name of intervention/drug, dosage form, administration, single dose, frequency of administration, and duration of intervention. (6) The outcome section has 19 fields, such as outcome name, endpoint/change value, direction of effect, result data, and data type (continuous or binary). Clinical data extraction requires clinical knowledge of TCM; hence, we trained data extractors before starting the work. We also employed two experienced reviewers to check all input data to ensure completeness and correctness.

#### 2.2.3. Data Standardization

Regarding standardization of the names of diseases, the names of TCMSDs and those of Western medicine were not unified and did not allow us to form a correspondence map. To create a unified standard, the names of diseases diagnosed by TCMSDs were used to frame the names of diseases diagnosed by Western medicine. With reference to the “11^th^ Revision of the International Classification of Diseases (ICD-11) [20], Classification and Code of TCM Diseases and Syndromes, and Clinical Terms of TCM diagnosis and Treatment [21],” we built a mapping table of TCMSD names and ICD-11 codes to construct the corresponding relationship between the TCMSD and the Western medicine names. We also standardized the TCM syndromes of TCMSDs to follow the “Classification and Code of TCM Diseases and Syndromes.” Regarding standardization of interventions, the interventions—either the treatment group or the control group—varied in name, dosage form, route of administration, single dose (and unit), and frequency of delivery, among other factors. For example, the intervention of acupuncture could be written as “acupuncture,” “acupuncture and moxibustion,” or “electro-acupuncture,” among others, and the Chinese herb medicine “Guipi decoction” could have different dosage forms such as pills, powder, granules, and capsules. We sorted out these cases and standardized different presentations using common terminologies at the data entry stage. We also applied similar standardization for the outcomes.

### 2.3. Database Development

MySQL [22] is an open-source database that is widely used and suitable for PHP, Python, and other languages. The MySQL database provides a variety of data types, including integer, floating-point, fixed-point, date and time, string, and binary [23]. The development of a database application program is convenient for users and enables access to and provides security to the data. We developed our database with Python 3.8 and MySQL 8 using Ubuntu 18. Several functional modules such as data input, managing, searching, and output were designed and implemented.

## 3. Results

### 3.1. Literature Search and Screening Results

The initial search returned 25,831 papers: 8,428 in Chinese (CNKI: 1,517, WanFang Data: 568, SinoMed: 6,237, and VIP: 106) and 17,403 in English (PubMed: 1,030, Cochrane Library (CENTRAL): 834, Web of Science Core Collection: 7,298, and Ebsco Medline: 8,241). Duplicates were filtered by NoteExpress and manually, resulting in 4,734 papers remaining for the next stage. The inclusion and exclusion criteria were applied to the titles and abstracts of the remaining, and 3,118 papers remained for full-text examination. We downloaded them and read their full text carefully, and finally, 1,600 papers of TCMSDs were included. As the main purpose of this paper was to verify the construction of the meta-evidence database, we chose the most recent five years of RCTs (total 405) for meta-evidence extraction.

### 3.2. Database Results

A total of 405 cases of TCMSD meta-evidence were collected with Excel tables and imported into the MED.

#### 3.2.1. Population

In the 405 cases of TCMSDs, the TCM diagnoses were mainly stomach stuffiness disease (125), epigastralgia (103), diarrhea disease (35), and constipation disease (18). These four TCM diagnoses accounted for 69% of all the included meta-evidence. The top five TCM syndromes were syndrome of Yang deficiency in the spleen and stomach (36), syndrome of cold and heat complex (16), syndrome of dampness and heat in the spleen and stomach (15), syndrome of spleen and stomach deficiency (15), and syndrome of disharmony of the liver and stomach (13). By comparing Western medicine diagnoses to TCM diagnoses, we found that the distribution was relatively uniform, and the top five occurrences were chronic atrophic gastritis of unknown etiology (65), functional dyspepsia (63), chronic superficial gastritis of unknown etiology (53), localized epigastric pain (33), and diarrhea (21) (Table 1).

#### 3.2.2. Interventions

TCM treatments were mainly herb medicines and Chinese patent drugs, such as banxiaxiexin decoction and its modifications, weifuchun tablets. Weiyan decoction, ziyinyangwei decoction, yiweishengjin decoction, etc., are also occasionally used in clinical use. They are usually combined with Western medicines of gastrointestinal motility drugs and prokinetic agents, such as domperidone, omeprazole, and mosapride citrate tablets (Table 2).

#### 3.2.3. Control Types

For TCMSDs, most of the included studies employed add-on tests (211 articles) or positive drugs as control (182 articles). Placebo control (3 articles), dose control (3 articles), and blank control (2 articles) were less common. (1) With respect to add-on trials, the patients both in the intervention group and control group were treated with the same baseline therapeutics, and the patients in the intervention group were further treated with TCM interventions. (2) Regarding positive controls, patients in the intervention group were treated with TCM, and those in the control group were treated with an effective routine approach.

#### 3.2.4. Outcomes

The outcomes of RCTs of TCMSDs include clinical efficacy measures (e.g., number of clinically ineffective, TCM syndrome scores, and number of relapses), safety measures (e.g., number of adverse events), and prognosis measures (e.g., number of relapses). (1) Clinical efficacy measures are quantitative indicators that can objectively describe the clinical treatment effects of interventions. (2) TCM syndrome scores can evaluate the severity and function of the human body. (3) Prognostic measures can reflect the development of disease recovery and outcome after intervention (Table 3).

### 3.3. Application Demonstration

We tested this database's functionality in a prototype ASR system (https://www.pymeta.com/cdss/). The fast EBM decision-making system, namely the TCM clinical evidence auto-analysis and visualization platform, was designed for rapid (even real-time) clinical and health decision-making (Figure 1). This system includes the MED, automatic meta-analysis, machine-based evidence-labeling, and result visualization modules, in which the MED has the key role of auto-SR support. Based on the TCM splenogastric disease meta-evidence, this platform allows an interesting and different process of SR (Figure 2). A typical application of this system starts from clinical problem (i.e., PICO) querying, matched RCTs (meta-evidence in this system) complete meta-analysis, and a systematic review in the background; the results of the effect and quality of evidence are present in the forms of text, tables, and figures. The platform acts on SR-based decision-making supporting in a fast and efficient way, it provides a new mode for evidence-based selection of drugs for TCMSDs from thousands of candidates.

## 4. Discussion and Conclusions

### 4.1. Main Findings

Meta-evidence is a form of evidence that can meet the needs of rapid evidence-based decision-making. It has the characteristics of standardization, structure, and machine-readability. In this study, we designed an extraction table to collect information of RCTs. All information was grouped in six sections: general information of evidence, source of evidence, clinical data of the study, RCT design, grouping and interventions, and outcomes. A total of 122 data fields within these sections were constructed as a detailed and structured data grid to cover all RCT information and transfer them into the MED. The meta-evidence was stored in a format that was easy for computer processing. As a sample of the MED, 405 cases of RCTs of TCMSDs were collected and extracted. For these studies, patients were diagnosed by TCM as suffering from stomach stuffiness disease and epigastralgia, and most of the TCM syndromes were Yang deficiency in the spleen and stomach, cold and heat complex, and dampness and heat in the spleen and stomach, among others. Regarding the interventions, herb medicine and Chinese patent drugs, such as banxiaxiexin decoction and weifuchun tablet, were the most commonly used. TCM medicines were usually combined with Western medicines of gastrointestinal motility drugs and prokinetic agents and tested in add-on trials. The outcomes of TCMSDs included clinical efficacy, safety, and prognosis measures, such as the number of clinically ineffective, TCM syndrome scores, number of adverse events, and number of relapses. The MED is an essential part of the ASR and rapid EBM decision-making system. The pre-extracted standardized data provide a strong basis for efficient data processing of ASRs. A prototype system of rapid EBM decision-making, namely the TCM clinical evidence auto-analysis and visualization platform, including the component of the MED of TCMSDs, passed the application test and proved the effectiveness and practicability of a MED.

In recent years, there have been many studies on automatic SRs assisted by computer [24], but most of them still adopt the semi-automatic method of “human-machine combination” [25]. Some meta-evidence similar data researches, such as the CISMeF metadata project, based on the Dublin core model, could describe the metadata of EBM resources [26], and Xu et al. [27] established an evidence-based medicine metadata experiment database. Another study [28] reported a web scraping algorithm developed by python language that can automatically extract metadata of published literature (such as title, abstract, keywords, year, author, and DOI). A brief comparison of automatic SR (and/or meta-analysis) and classical manual SR is shown in Table 4.

### 4.2. Limitations and Outlook

MED-TCMSD was constructed and tested for advancement. However, there are some details that should be improved in the future. (1) Only five years of TCMSD RCT data were included in this sample database. We plan to process the remaining literature in the future. (2) All the extraction work of the meta-evidence was completed by experienced researchers, which consumed substantial manpower and time resources. We are searching for efficient and sustainable solutions, such as computer-aided technologies and crowdsourcing collaboration to replace the current, inefficient manual methods.

### 4.3. Conclusions

Rapid decision-making based on automatic SR techniques is an interesting direction of evidence-based medicine development. ASR techniques need to be supported by more efficient databases than the classical forms of EBM databases (such as RCT, SR, and CPG). Our new EBM database is highly standardized, structured, and machine-readable, which precisely meets all the requirements of ASRs. A sample of this kind of database, MED-TCMSD, was completed, which has a key role in the ASR and rapid decision-making system. We believe that the meta-evidence approach is a good solution for ASR databases, and the method of constructing MED-TCMSD can be further applied in the development of MEDs for other diseases.

## Figures and Tables

**Figure 1:** Overview of the TCM Clinical Evidence Auto-analysis and Visualization Platform. (This figure shows the main parts of the platform, the upper input area of PICO, and results area below it, which includes left side of outcoms lists and right side of graphs of PICO-network and evidence-map. The included RCTs show in the bottom table).

**Figure 2:** Evidence map based on MED-TCMSD. (Evidence map is the common visualization form of evidence-based decision-making supporting, which present effect (x-axis) and quality (y-axis) of multievidence for the same clinical problem).

**Table 1:** Population of included TCMSD RCTs.

TCM diagnosis	Number	TCM syndrome	Number	Western medicine diagnosis	Number
Stomach stuffiness disease	125	Syndrome of Yang deficiency in spleen and stomach	36	Chronic atrophic gastritis of unknown etiology	65
Epigastralgia	103	Syndrome of cold and heat complex	16	Functional dyspepsia	63
Diarrhea disease	35	Syndrome of dampness and heat in the spleen and stomach	15	Chronic superficial gastritis of unknown etiology	53
Constipation disease	18	Syndrome of spleen and stomach deficiency	15	Localized epigastric pain	33
Abdominal pain	6	Syndrome of disharmony of the liver and stomach	13	Diarrhea	21
Regurgitation disease	6	Syndrome of spleen and stomach qi deficiency	9	Functional constipation	16
Acid regurgitation	4	Syndrome of stagnant heat in the liver and stomach	9	Rheumatoid arthritis	15
Dysentery	2	Syndrome of liver depression and spleen deficiency	8	Gastric ulcer	11
Vomiting	1	Syndrome of qi stagnation due to spleen deficiency	5	Gastritis caused by *H. pylori*	8
Epigastric upset	1	Syndrome of dampness and heat	4	Symptomatic diarrhea	7

**Table 2:** Interventions of included TCMSD RCTs.

Intervention/drug name	Number	Control/drug name	Number
Modified banxiaxiexin decoction	16	Domperidone	24
Banxiaxiexin decoction	7	Omeprazole	21
No. 1 Weiyan decoction	3	Weifuchun tablets	11
Ziyinyangwei decoction	2	Conventional therapy	8
Yiweishengjin decoction	2	Mosapride citrate tablets	8
Yiqihuoxue recipe	2	Montmorillonite powder	6
Xiangsha liujunzi tang	2	Cisapride	6
Xiaopi granules	2	Vitamin tablets	5
Modified sini powder	2	Rabeprazole	4
Qizhiweitong granules	2	Routine nursing	4
Buzhongyiqi decoction	2	Trimebutine maleate tablets	3

**Table 3:** Outcomes of included TCMSD RCTs.

Name of outcome measure	Number
Number of clinically ineffective	345
Total number of adverse events	81
TCM syndrome scores (epigastralgia)	77
TCM syndrome scores (fullness)	59
TCM syndrome scores (anorexia)	54
TCM syndrome scores (belching)	47
TCM syndrome scores (total)	43
Number of relapses	40
Serum level (motilin)	30
Symptom scores (stomachache)	30
Serum level (gastrin)	29
Number of adverse events (diarrhea)	26
TCM syndrome inefficiency number	22
TCM syndrome scores (nausea and vomiting)	22
Number of adverse events (dizzy)	20
TCM syndrome scores (loose stool)	20
TCM syndrome scores (sour regurgitation)	20
No improvement of gastroscopy	18
Number of adverse events (rash)	17
TCM syndrome scores (mental fatigue)	17
Number of *H. pylori* positive	16
Symptom scores (fullness)	14
Serum level (IL-6)	14
TCM syndrome scores (noisy stomach)	14
Symptom scores (belching)	13
Number of adverse events (nausea)	13
Number of adverse events (dry mouth)	13
Number of adverse events (astriction)	13
Symptom scores (anorexia)	12
Number of *H. pylori* negative	11

**Table 4:** Automatic SR and manual SR.

SRs process	Automatic SR	Manual SR
Literature retrieval	PICOS precise retrieval in multiple databases, subject auto push periodically	Manual indexing and searching in multiple databases
Literature screening	RCT classification based on machine learning	Manual screening based on experience
Data extraction	Full or semi-automatic extraction of PICO information from the paper	Manual extraction and fill the datasheet
Data analysis	Automatic meta-analysis based on modules of statistics and meta-evidence databases	Manual data entry and setup parameters in SR software
Evidence quality assessment	Full or semi-automatic evidence quality assessment	Manual assessment based on expertise and experience

## Data Availability

The data used to support the findings of this study are included within the article. Data are available from the corresponding author upon request.

## Abbreviations

TCMSDs: Traditional Chinese medicine splenogastric diseases
MED-TCMSD: Meta-evidence database of traditional Chinese medicine splenogastric disease
TCM: Traditional Chinese medicine
RCTs: Randomized controlled trials
SRs: Systematic reviews
IBS: Irritable bowel syndrome
EBM: Evidence-based medicine
CPG: Clinical practice guideline
ASRs: Automatic systematic reviews
VBA: Visual basic for applications
ICD-11: 11th revision of the international classification of diseases
PICOS: Patient/population, intervention/exposure, comparison/control, outcome, study design
IL-6: Interleukin-6.
